This article has been retracted.

# Direct Detection of Antibiotic Resistance in Chinese *Helicobacter pylori* Clinical Isolates by Sequencing-Based Approach

**DOI:** 10.1155/2022/6436256

**Published:** 2022-04-15

**Authors:** Lixia Tian, Yi Yao, Li Yin, Lanxiang Wang, Ze An, Lin Kang, Chenglin Ru, Jinping Li

**Affiliations:** ^1^Department of Emergency Medicine, The Eighth Medical Center, Chinese PLA General Hospital, Beijing, China; ^2^Department of Gastroenterology, The Eighth Medical Center, Chinese PLA General Hospital, Beijing, China; ^3^Western Medical District of Chinese PLA General Hospital, Beijing, China; ^4^Department of Xiangshan Road Clinic, The Eighth Medical Center, Chinese PLA General Hospital, Beijing, China; ^5^State Key Laboratory of Pathogen and Biosecurity, Beijing Institute of Microbiology and Epidemiology, Beijing, China; ^6^Department of Ultrasound, The Eighth Medical Center, Chinese PLA General Hospital, Beijing, China; ^7^Department of Gastroenterology, The First Medical Center, Chinese PLA General Hospital, Beijing, China

## Abstract

**Objective:**

The detection of *Helicobacter pylori* mutations that result in antimicrobial resistance can serve as a guideline of antimicrobial therapeutics and probably prevent the failure of clinical treatments. Evaluating the potential of Sanger sequencing to identify genetically resistant determinants in *Helicobacter pylori* clinical isolates will be important.

**Methods:**

180 cultured strains have been tested using agar dilution for antibiotic susceptibility. NCBI BLAST was used to perform genotypic analysis on the sequencing data. Sanger sequencing was evaluated as an alternative method to detect resistant genotypes and susceptibility.

**Results:**

By the conventional E-test, resistance to levofloxacin, amoxicillin, metronidazole, and clarithromycin was 67.3%, 15.1%, 96.4%, and 25.5%, respectively. In contrast, tetracycline had no resistance. Resistance to multiple drugs was observed in 8.12% of the strains. The genetic determinants of resistance to CLA was 23s rRNA, the determinants of resistance to amoxicillin was Pbp1, the determinants of resistance to metronidazole was rdxA, and the determinants of resistance to levofloxacin were GyrA and GyrB. However, there was no association of resistance in tetracycline.

**Conclusion:**

We found increased rates of metronidazole antibiotic resistance, highlighting the necessity for alternative therapies and periodic evaluation. Sanger sequencing has proved to be highly effective and holds the potential to be implemented in policies catering to local treatments.

## 1. Introduction

Widespread use of antibiotics has had a profound impact on the whole life of bacteria [1]. Many pathogen strains have become resistant to antibiotics and even multidrug resistance [2]. It has been proven that drug resistance can make the efficacy of many existing drugs and decrease and disappear, leading to more than 700,000 deaths in one year [3, 4], which is one of the greatest public health issues [5, 6].

According to the WHO, *Helicobacter pylori* can cause many gastrointestinal disorders such as gastritis, peptic ulcers, and gastric cancer [7], which is the main threat to human health [8]. However, the efficacy of current therapies for *Helicobacter pylori* was dramatically decreasing because of the increased antibiotic resistance [9]. Therefore, many conferences for *Helicobacter pylori* treatments have been held to deal with antibiotic resistance [10, 11]. In developed countries, the infection rate of *Helicobacter pylori* ranges from 25% to 50%, whereas in developing countries, the rate is up to 80%. The infection rate in China is also numbered as high as 56.2% [12]. The widespread use of eradication therapeutic regimens, consisting of at least two antimicrobial agents, has recently shown that the resistance of *Helicobacter pylori* to antimicrobial agents such as clarithromycin, fluoroquinolones like levofloxacin, and metronidazole shows an increasing trend year by year.

Routine *Helicobacter pylori* sensitivity tests are very difficult under current conditions because *Helicobacter pylori* needs a nutrient-rich, selective medium [13]. Therefore, it is particularly important to find a timely and accurate method to diagnose drug resistance in the clinical treatment of *Helicobacter pylori*. Molecular biology techniques can identify the molecular mechanisms of various antimicrobial agents [14–16]. And a molecular testing strategy also can comprehensively assess the multifaceted information associated with *Helicobacter pylori* therapy in one test [17]. It can not only assist clinicians in issuing individualized solutions for *Helicobacter pylori* treatment for different patients, but also help to promote the progress of research on the mechanism of molecular treatment for *Helicobacter pylori* [18, 19].

Based on the abovementioned, we characterized the resistance rate of amoxicillin, clarithromycin, metronidazole, levofloxacin, and tetracycline from *Helicobacter pylori*, which are the five antibiotics commonly used in *Helicobacter pylori* treatments. We also use Sanger sequencing, which is the most common approach to determine the mutations conferring resistance, to detect resistant genotypes, determine susceptibility, and evaluate the correlation between their phenotypes and genotypes.

## 2. Materials and Methods

### 2.1. Sample Collection

The study included 160 *Helicobacter pylori* treatment naive outpatients (80 in 2014-2015 and 80 in 2018-2019). They had an esophagogastroduodenoscopy examination at Chinese PLA General Hospital in 2014-2015 and 2018-2019. During the endoscopic procedure, gastric biopsy specimens were taken, then we inoculated them on a *Helicobacter pylori*-selective plate [20]. After performing a series of biochemical reactions using catalase, oxidase, urease, and stained gram, *Helicobacter pylori* colonies, which were circular, clear, convex, and purple, were identified under light microscopy observation [21]. All procedures were incubated at 37°C and performed in microaerophilic conditions (10% O_2_, 5% CO_2_, and 85% N_2_).

### 2.2. Phenotypic Characterization of Antimicrobial Susceptibility

The agar dilution assay was used to define the antibiotic susceptibility phenotype. Five antibiotics such as amoxicillin, metronidazole, clarithromycin, tetracycline, and levofloxacin were used in this experiment. *Helicobacter pylori* were cultured for 72 h, then the antibiotic MIC was inferred using *Helicobacter pylori* strain 26695 as the control. Antibiotic MIC is the minimum inhibitory concentration of antibiotics, which is always used to define the antibiotic susceptibility phenotype. When the MIC of metronidazole exceeded 8 mg/L, tetracycline and levofloxacin exceeded 1 mg/L, clarithromycin exceeded 0.25 mg/L, and amoxicillin exceeded 0.125 mg/L, it was defined as antibiotic resistance [22, 23].

### 2.3. Genotype Analysis of Antibiotic Susceptibility

Snippy v.3.2 and Gubbinsv2.3.4 were used to core SNP alignment and predict recombinant regions aimed to assess the relatedness between *Helicobacter pylori* strains. The antibiotic susceptibility genotypes, such as GyrA and GyrB for levofloxacin, 23S rRNA for clarithromycin, Pbp1 for amoxicillin, RdxA for metronidazole, and 16S rRNA for tetracycline were assessed. Variant identification, summarization, and assessment were performed for the association with the resistance phenotype. Besides, Phandango was used to perform the phenotypic resistance patterns to heat maps and antibiotic resistance.

### 2.4. Statistical Analysis

SPSS 17.0 statistical software was used for statistical analysis. The quantitative data were expressed as the mean ± standard deviation (mean ± SD). The *t*-test was used for comparison between two groups, and *P* < 0.05 was considered a statistically significant difference.

## 3. Results

As the antibiograms of 160 isolates from Beijing in Table 1, we noted the resistance rates of metronidazole, levofloxacin, clarithromycin, amoxicillin, and tetracycline decreased in the order of 96%, 67%, 25%, 15%, and 0, respectively, and 14 strains were susceptible to all (Figure 1).

### 3.1. *Helicobacter pylori* Antibiotic Susceptibility in Beijing

The proportion of single-drug resistance was 21.8% among all drug-resistant isolates, and all were metronidazole resistant. The proportion of multi-drug resistance was 76.4%. Among all clinical isolates, the dual resistance rate to levofloxacin + metronidazole was 40%, and the dual resistance rate to metronidazole + clarithromycin was 7.3%. Triple resistance to amoxicillin + levofloxacin + metronidazole was 9.1% and to clarithromycin + levofloxacin + metronidazole was 18.2% (Figure 2).

### 3.2. Comparison between Genotypes and Phenotypes

After the comparison of the phenotypes and the corresponding genotypes, we found that the determinants of resistance to levofloxacin were GyrA and GyrB, the determinant of resistance to amoxicillin was Pbp1, the determinant of resistance to metronidazole was rdxA, and the determinant of resistance to CLA was 23s rRNA (Figure 3). There was complete concordance between genotype and phenotype for clarithromycin and concordance for levofloxacin and amoxicillin (Table 2).

## 4. Discussion

Our study suggests that the resistance of *Helicobacter pylori* isolates may be due to the extensive use of antibiotics, especially metronidazole, clarithromycin, and amoxicillin. For example, the resistance to metronidazole in *Helicobacter pylori* clinical isolates may be because of prescriptions for parasitic infections, pelvic inflammation, or dental infections [24–26]. Furthermore, resistance of drug-resistant *Helicobacter pylori* to levofloxacin is similarly high, which may be caused by using levofloxacin to treat urinary and respiratory tract infections [27–29].

As high MIC values in metronidazole and clarithromycin resistant strains are associated with resistance patterns in vivo, they are perhaps potential markers for predicting curable rates. As no plasmids were found in all strains, indicating that *Helicobacter pylori* resistance is based on mutations, it also inspired us to think that detection of point mutations in the genome can be used to identify *Helicobacter pylori* resistance.

Molecular susceptibility testing is becoming the ideal for detecting drug resistance in *Helicobacter pylori* clinical isolates due to greater speed as well as greater accuracy [30]. Sanger sequencing may not have an impact on strain resistance [31–33]. We thus need to explore new approaches like phenotypic characterization of antimicrobial susceptibility and genotype analysis of antibiotic susceptibility [34, 35]. Furthermore, regular assessment and alternative therapies are also important to control the resistance status. This study's novelty lies in the reporting of resistance patterns of *Helicobacter pylori* clinical isolates, providing an overview of the current state of antibiotic resistance, which can guide the elimination of *Helicobacter pylori*.

However, this study also has partial limitations. First of all, the samples in this study were all patients from a hospital, which cannot reflect *Helicobacter pylori* patterns in the general population. Second, the sample size of partial resistance to antibiotics in this study was small, and the strength of the association was only associated with few or no resistant strains, such as amoxicillin and TET. Third, the present study was conducted at the *in vitro* level, and the commonly used antibiotic resistance rates revealed by the study data were not completely accurate, and clinical trials are needed for further validation.

## 5. Conclusion

This findings show that *Helicobacter pylori* had resistance to antibiotics and was also likely to be pathogenic and virulent. In addition, molecular susceptibility testing that detects genetic determinants associated with drug resistance can be used in detection tests for *Helicobacter pylori* drug resistance. However, due to various limitations, it is necessary to continue to expand the sample size and continue clinical trials in the future.

## Figures and Tables

**Figure 1:** The range and distribution of MIC values for each antibiotic. A resistance profile with the highest prevalence of resistance to metronidazole 96.4% (95% CI, 87.5–99.6), followed by levofloxacin 67.3% (95% CI, 53.3–79.3), clarithromycin 25.5% (95% CI, 14.7–39), and amoxicillin 15.1% (95% CI, 10.1–31.9).

**Figure 2:** Comparisons of multiple antibiotic resistance rates. In 2014-2015, 14.6% of *Helicobacter pylori* isolates were susceptible to all antibiotics, with 33.7%, 28.3%, 16.7%, 6.2%, 0.3%, and 0.3% being isolate resistance, double resistance, triple resistance, quadruple resistance, quintuple resistance, and sextuple resistance, respectively. In 2018-2019, 9.4% of *Helicobacter pylori* isolates were susceptible to all antibiotics, with 27.6%, 28.4%, 24.9%, 7.3%, 2.3%, and 0.1% being isolate resistance, double resistance, triple resistance, quadruple resistance, quintuple resistance, and sextuple resistance, respectively.

**Figure 3:** Comparison between antibiotic susceptibility genotypes and phenotypes. Maximum likelihood phylogenetic trees were built for the resistance patterns of each antibiotic and their corresponding genetic determinants. Dark blue and red rectangles represented sensitive and resistant patterns. Green and grey rectangles denote mutations and no mutation, respectively.

**Table 1:** Resistance pattern of *Helicobacter pylori* strains.

Resistance pattern	Number of strains
All susceptible	14
All resistance	0
Levofloxacin	108
Amoxicillin	24
Metronidazole	154
Clarithromycin	41
Tetracycline	0
Mono resistance	
Levofloxacin only	13
Amoxicillin only	5
Metronidazole only	0
Clarithromycin only	5
Tetracycline only	12
Multiple resistance	
Levofloxacin + metronidazole	64
Clarithromycin + metronidazole	12
Amoxicillin + levofloxacin + metronidazole	15
Clarithromycin + levofloxacin + metronidazole	29

**Table 2:** Comparison between genotypes and phenotypes.

Antibiotics	Phenotypic	Genotypic		Kappa values
		Yes	No	
Metronidazole	Yes	139	15	0.279
	No	2	4	
Levofloxacin	Yes	91	17	0.705
	No	5	47	
Clarithromycin	Yes	35	5	0.848
	No	4	116	
Amoxicillin	Yes	17	8	0.727
	No	2	134	

## Data Availability

The data used to support this study are available from the corresponding author upon request.
